# Effects of Seamless Operating Room Nursing Combined with Multistyle Health Education on the Psychological State, Rehabilitation Quality, and Nursing Satisfaction in Patients with Internal Fixation of Femoral Fracture

**DOI:** 10.1155/2022/5196363

**Published:** 2022-04-05

**Authors:** Qingyan Liu, Juan Wang, Jie Han, Tongyang You, Lijuan Li

**Affiliations:** The Operating Room, the Affiliated Hospital of the Southwest Medical University, 25 Taiping Road, Luzhou 646000, Sichuan, China

## Abstract

**Objective:**

To explore the effects of seamless operating room nursing combined with multistyle health education on the psychological state, rehabilitation quality, and nursing satisfaction in patients with internal fixation of femoral fracture.

**Methods:**

Eighty patients who received internal fixation of femoral fracture in our hospital (November 2020–November 2021) were chosen as the research objects, and their clinical data were retrospectively analyzed. They were divided into experimental group and control group according to the sequence of hospital admission. In perioperative period, the control group received routine nursing measures and the experimental group received seamless operating room nursing combined with multistyle health education. The patients' psychological state, rehabilitation quality, and nursing satisfaction after intervention were compared between the two groups.

**Results:**

Compared with the control group, the experimental group achieved remarkably lower score of Profile of Mood States (POMS) after nursing (*p* < 0.001). The experimental group had much higher cognitive level scores, Harris hip score (HHS), Functional Independence Measure (FIM) score, and nursing satisfaction score in comparison with the control group (*p* < 0.05). In perioperative period, the experimental group had much lower total incidence of complications in comparison with the control group (*p* < 0.05).

**Conclusion:**

Seamless operating room nursing combined with multistyle health education, as an effective measure to improve the rehabilitation quality of the patients with internal fixation of femoral fracture, has better effects on improving the patients' psychological state and reducing complications in perioperative period in comparison with the routine nursing intervention. Further studies are conducive to providing a better solution for the patients with internal fixation of femoral fracture.

## 1. Introduction

With the frequent occurrence of traffic accidents, falling accidents, and other dangerous events in recent years, the patients suffering from femoral fracture has been increasing year by year in China [1]. Internal fixation of femoral fracture is a commonly used surgical treatment for femoral fracture, and its purpose is to restore the normal function of limbs to the maximum extent by reconstructing the anatomical structure of bones [2, 3]. Most patients with femoral fracture are middle-aged and elderly people, who are complicated with multiple chronic diseases and always develop negative emotions before the surgery, so there are many difficulties when performing the surgery [4]. Besides, the surgery may aggravate the patients' stress responses, and inadequate preparation before the surgery may lead to the occurrence of hazard events during surgery and unsatisfactory surgery effect. Therefore, implementing operating room nursing is crucial to enhance the treatment effect of the internal fixation of femoral fracture [2, 5]. With the continuous development of medical models, seamless operating room nursing has been considered as a comprehensive and meticulous nursing intervention model [4]. Seamless operating room nursing has remarkable effects on helping the patients to go through their perioperative period smoothly, reducing their stress responses, and promoting their physical and mental health. The efficacy of seamless operating room nursing has been confirmed in the excision of gastrointestinal tumor, in the intubation of total knee joint in the patients with bone tumor and in the treatment of craniocerebral injury [6–8]. Multistyle health education can provide the patients with diversified clinical health education and more choices (like holding health knowledge lectures, distributing video brochures, and conducting education through video and in WeChat group), so as to ensure the targeted and timely health education [9]. At present, there are few studies exploring the effects of seamless operating room nursing combined with multistyle health education on the perioperative intervention in patients with internal fixation of femoral fracture. This study aims at filling in this blank and providing more evidence-based bases for the patients.

## 2. Materials and Methods

### 2.1. General Data

Eighty patients who received internal fixation of femoral fracture in our hospital (November 2020–November 2021) were chosen as the research objects. They received related clinical examinations after admission. This study conformed with the *Declaration of Helsinki (2013)*[10].

### 2.2. Inclusion and Exclusion Criteria

Inclusion criteria were as follows: ① the patients' surgical indications were definite, and the patients had underwent internal fixation of femoral fracture; ② the patients had normal communication and comprehension abilities; ③ the patients' clinical data were complete.

Exclusion criteria were as follows: ① the patients had the history of hip trauma or congenital hip disease; ② the patients were complicated with severe cardiovascular and cerebrovascular disease or endocrine disease; ③ the patients had severe hearing impairment or visual disorder.

### 2.3. Methods

All the patients in the two groups received internal fixation of femoral fracture and combined spinal-epidural anesthesia. The patients were injected with 1–5 *μ*g of sufentanil through intravenous drip (manufacturer: Yichang Humanwell Pharmaceutical Co., Ltd.; NMPA Approval No. H20030199; specification: 5 ml:375 *μ*g). After the drug worked, the diseased limb was drawn and the upper body was kept in supine position. Then, the epidural puncture and the puncture in subarachnoid space were performed. When the cerebrospinal fluid flowed fluently, the patients were given 10–13 mg mixed liquids of 2 ml ropivacaine injection (0.75%; manufacturer: Jiabo Pharmaceutical Co., Ltd.; NMPA Approval No. H20113381; specification: 10 ml:75 mg) and 1 mL sodium chloride (0.9%). After finishing the anesthesia, the patients' vital signs were monitored. The patients in the control group received routine nursing measures in perioperative period. To be specific, the nursing staff visited the patients before surgery, instructed them to make preoperative preparation, and informed them of postoperative matters needing attention. After being sent to the operating room, the patients received anesthesia and surgery. After the surgery, the patients were sent to the ward and the nursing staff conducted the connection work with ward nurses [11]. After 6 hours of the surgery, the patients received the liquid diet. According to the patients' personal intentions, the nurses guided them to move their bodies. The nursing staff pacified the patients' and their families' emotions and repeatedly advised the patients to have adequate rest time.

The experimental group received seamless operating room nursing combined with multistyle health education in perioperative period. The specific seamless operating room nursing measures were as follows: ① the seamless operating room nursing groups were established. The nursing staff were comprehensively evaluated in the aspects of nursing experience, working ability, and positional title. The hierarchical management was implemented to quantify and clarify the responsibility and duty of each nursing staff. The nursing staff were divided into several groups, with 1 head nurse and 4 nurses in each group. The head nurse presided over the shifting of duty, inspected the patients' conditions in wards, collected written reports, and explained relevant matters needing attention. A flexible scheduling program was developed according to actual situation, so as to ensure continuous and seamless nursing work. ② Preoperative nursing: all group members visited the patients together, and the circulating nurses introduced the responsibilities of different nurses to every patient. All nurses interacted with the patients to establish a good nurse-patient relationship. The circulating nurses were responsible for the patients' psychological counseling, so as to lead the patients to maintain a good psychological state and eliminate inner fears and tensions. ③ Intraoperative nursing: after successful induction of anesthesia, the patients' temperature, blood pressure, heart rate, and other indicators were closely monitored in surgery, and the nursing staff cooperated with surgeons to complete the surgery. During the surgery, the changes of patients' vital signs were closely observed, and then they were sent back to wards by the circulating nurses after meeting awakening conditions. The nursing staff should hand over the patients' information carefully. The ward nurses should accurately grasp the patients' intraoperative conditions and the indications requiring attention after surgery, for example, blood filling at the end of limbs, blood circulation, fluctuating pain, and pyogenic infection in surgical wound. The surgery nurses should revisit the patients one day after surgery and carefully check the patients' postoperative indications and the implementation of nursing measures. The nursing staff should take the initiative to carry out appropriate communication with patients, so as to make them fully understand their own conditions and surgery.

The specific contents of multistyle health education were as follows: ① the professional orthopedic experts were invited to conduct lectures about health knowledge, so as to comprehensively and systematically explain the knowledge of femoral fracture (including pathogenesis, treatment methods, and clinical nursing) and the postoperative matters needing attention to patients. During the lecture, the patients were encouraged to ask questions and the professional physicians answered the questions to eliminate the patients' doubts and improve their cognition toward their diseases. ② The nursing staff distributed health brochures to patients, which included the causes, common symptoms, disease types, and inducing factors of femoral fracture. The nursing staff carefully introduced the contents in the brochure to the patients, instructed them to read the brochure in detail, and guided them to understand the preventive measures, treatment methods, nursing approaches, and postoperative matters needing attention of the disease. ③ Video education: various forms of microvideos were produced to introduce the knowledge of femoral fracture and operation procedures of internal fixation by explaining specific cases. The patients were required to watch different videos of health education according to their conditions. The easy-to-understand and vivid videos could strengthen the patients' knowledge of their own disease. ④ A WeChat group was formed, and the members included patients, nursing staff, and physicians. The professional knowledge of femoral fracture was sent to the WeChat group to make the patients master the correct specialized knowledge. The patients were required to give a brief description of their physical conditions and were supervised and urged to do rehabilitation exercise if their body conditions allowed. The WeChat group was a relaxed, normative, and civilized communication platform, where the nursing staff and physicians answered the patients' questions and provided service to them.

### 2.4. Observational Indexes

The Profile of Mood States (POMS)[12] questionnaire was adopted to assess the patients' mood states after nursing. This profile included 7 dimensions of fatigue, vigor, tension, confusion, and so on, with 40 items in total. Negative emotion score minus positive emotion score was the final score. Higher scores indicated deeper mood states.

The questionnaire of inpatients' clinical satisfaction made by our department was adopted, and this questionnaire included the patients' satisfaction on nursing skills, attitude, and effect. The total score was 100 points; 85–100 points indicated full satisfaction; 70–84 points indicated satisfaction; 55–69 points indicated general satisfaction; 0–54 points indicated dissatisfaction.

Harris hip score (HHS) [13] and Functional Independence Measure (FIM) [14] were adopted to assess the patients' rehabilitation quality after intervention. FIM included the pain level (44 points), functioning level (47 points), joint range of motion (5 points), and limb deformity (4 points). The total HHS was 100 points, and higher scores indicated better hip joint function. The total score of FIM was 126 points, and higher scores indicated better motor and cognitive function and higher independence.

The questionnaire of cognitive level designed by our hospital was adopted to assess the patients' cognition on the disease, self-nursing, and treatment, and the score of each item was 0–5 points. Higher scores indicated higher cognitive levels.

The complications occurred in perioperative period were recorded and counted. The complication types included fracture nonunion, pressure ulcer, deep venous thrombosis of lower extremities, and joint stiffness.

### 2.5. Statistical Treatment

The professional statistical software SPSS26.0 was adopted for data processing, and GraphPad Prism 7 (GraphPad Software, San Diego, USA) was used to draw graphs of the data in this study. The count data were tested by X^2^ and expressed by (*n*(%)). The measurement data were tested by *t* and expressed by mean ± SD. When *P* < 0.05, the differences were considered statistically significant.

## 3. Results

### 3.1. Clinical Data

No remarkable difference was observed in sex ratio, average course of disease, causes of injury, types of fracture, and other general data (*p* > 0.05; Table 1).

### 3.2. Psychological State

Compared with the control group, the experimental group achieved remarkably lower POMS score after nursing (*p* < 0.001; Figure 1).

### 3.3. Cognitive Level

The experimental group had much higher cognitive level scores in comparison with the control group (*p* < 0.05; Table 2).

### 3.4. Rehabilitation Quality

The experimental group had much higher HHS and FIM score after surgery in comparison with the control group (*p* < 0.001; Table 3).

### 3.5. Nursing Satisfaction Score

The experimental group had much higher nursing satisfaction score in comparison with the control group (*p* < 0.001; Figure 2).

### 3.6. Complications in Perioperative Period

In perioperative period, the experimental group had much lower total incidence of complications in comparison with the control group (*p* < 0.05; Table 4).

## 4. Discussion

Accidental falls and the hit by heavy objects are the main causes of femoral fracture, whose clinical manifestations are obvious swelling and pain at the fracture site and even distortion and angulation deformity in severe cases [15]. Internal fixation of femoral fracture is the main treatment. After the fixation, the patients' bones can be effectively reset and the normal physiological function at the fracture site can be recovered. However, the patients may develop muscular atrophy, lower extremity venous thrombosis, and other complications after surgery, affecting their recovery [16]. Therefore, this study, based on the previous clinical nursing experience, implemented seamless operating room nursing combined with multistyle health education in patients with internal fixation of femoral fracture, so as to further explore the effects of this nursing plan on disease.

The operating room is an important place for diagnosis, treatment, and rescue, and surgical operation is a great physical and psychological stressor for patients. In the operating room, the patients not only face the trauma brought by surgical operations but also suffer from negative emotions, which affect the effect of surgery and their postoperative recovery to a certain extent [17]. As people's self-protection awareness has increased in recent years, the patients have higher requirements for surgical comfort, as well as the involvement and selectivity in treatment. Superior operating room nursing not only greatly eliminates the patients' preoperative fear and nervousness but also enhances the efficiency and success rate of surgery. As a new, high-quality, and modern nursing model, the seamless operating room nursing has gradually demonstrated its advantages and characteristics in clinical practice and has become a new breakthrough and a model of modern service management [18]. Seamless operating room nursing adheres to the philosophy of “putting people first,” implements the service concept of “one-stop service” in the work, and attempts to benefit patients by putting them at the center. The nursing efficacy of seamless operating room nursing has been confirmed in resection of gastrointestinal tumors, trigeminal nerve microvascular decompression, and other surgeries. According to clinical studies [19], the fracture and surgery are likely to damage the nutritional vessels and affect the blood supply to the distal fracture segment. As a result, the patients suffer from blood circulatory disorder and develop many complications. Some scholars [20] have pointed out that the incidence of surgical complications in the patients who have underwent orthopedic surgery can reach 60% without any preventive measures. Health education is an effective measure to enhance patients' cognition of disease and self-management ability, but the patients' actual requirements cannot be guaranteed under the conventional indoctrination health education, resulting in uneven effects of clinical education [21]. Multistyle health education provides patients with the lively orthopedic health education by utilizing pictures, audios, and videos and integrating different health education forms (such as video education, health knowledge lecture, and WeChat groups), so as to ensure the pertinence and effectiveness of health education.

According to the study results, the experimental group had better mood states after receiving joint intervention (*p* < 0.001), and the reasons behind were speculated as follows. During the seamless operating room nursing, all the nurses proactively participated in the nursing service and conducted health education and psychological intervention according to the patients' specific conditions before surgery, which greatly reduced the patients' preoperative fear and tension and improved their mental states [22]. In terms of complications in perioperative period, the experimental group had much lower total incidence of complications in comparison with the control group (*p* < 0.05). In this study, fracture nonunion and deep venous thrombosis of lower extremities are the common complications, indicating that the nursing staff should sufficiently prevent the occurrence of these complications. In terms of the rehabilitation quality, the joint intervention model, by conducting the education and publicity for the patients with femoral fracture, is conducive to improving the patients' understanding of the disease and enhancing their self-management ability. As a result, this intervention model can accelerate the recovery of hip joints and improve the rehabilitation quality. Besides, the nursing satisfaction in the experimental group was much higher compared with the control group (*p* < 0.05). The seamless operating room nursing was patient-centered and aimed at benefiting the patients and safeguarded the patients' rights and interests in all aspects. The responsibility, caring, and enthusiasm presented by the medical and nursing staff during the nursing process were conducive to establishing a good patient-nurse relationship and improving the patients' satisfaction with the nursing. This study result basically coincided with the report of Eriksson et al. [23].

Because of the limitations of the study conditions, the study objects only included 80 patients and the sample size was small, which inevitably had an impact on final results. Besides, the seamless operating room nursing, requiring the coordination between different departments, had heavy workload and difficulty in operation.

## Figures and Tables

**Figure 1:** Comparison of the POMS score (mean ± SD). Note: the abscissa indicated the experimental group and the control group, and the ordinate indicated POMS score (points); the POMS scores of the experimental group and the control group were (11.65 ± 1.81) points and (20.08 ± 2.45) points, respectively; ^*∗*^ indicated a remarkable difference in the POMS scores between the two groups (*t* = 17.503, *p* < 0.001).

**Figure 2:** Comparison of the nursing satisfaction score (mean ± SD). Note: the abscissa indicated the experimental group and the control group, and the ordinate indicated the nursing satisfaction score (points); the nursing satisfaction scores in the experimental group and the control group were (82.55 ± 5.22) points and (63.30 ± 7.02) points, respectively; ^*∗*^ indicated a remarkable difference in the nursing satisfaction scores between the two groups (*t* = 13.917, *p* < 0.001).

**Table 1:** Comparison of clinical data.

Items	Experimental group	Control group	X^2^/*t*	*p*
Sex			0.050	0.823
Male/female	21/19	22/18		
Average age (mean ± SD, years old)	55.80 ± 5.47	56.10 ± 5.49	0.245	0.807
Average course of disease (mean ± SD, d)	3.60 ± 1.68	3.83 ± 1.71	0.607	0.546
Causes of injury				
Hit by heavy objects	11 (27.50)	14 (35.00)	0.524	0.469
Accidental fall	26 (65.00)	24 (60.00)	0.213	0.644
Others	3 (7.50)	2 (5.00)	0.213	0.644
Types of fracture				
Type II	11 (27.50)	9 (22.50)	0.267	0.606
Type III	13 (32.50)	14 (35.00)	0.056	0.813
Type IV	13 (32.50)	15 (37.50)	0.220	0.639
Type V	3 (7.50)	2 (5.00)	0.213	0.644
Affected side			0.050	0.823
Left side	21 (52.50)	22 (55.00)		
Right side	19 (47.50)	18 (45.00)		
Place of residence			0.202	0.653
Urban areas	17 (42.50)	19 (47.50)		
Rural areas	23 (57.50)	21 (52.50)		

**Table 2:** Comparison of cognitive level scores (mean ± SD).

Group	n	Knowledge related to disease	Knowledge related to self-nursing	Knowledge related to treatment
Experimental group	40	4.03 ± 0.86	3.70 ± 1.09	3.48 ± 1.24
Control group	40	2.93 ± 0.83	2.08 ± 0.80	2.85 ± 0.89
*t*		5.821	7.578	2.610
*P*		<0.001	<0.001	<0.05

**Table 3:** Comparison of the rehabilitation quality after surgery (mean ± SD).

Group	n	HSS	FIM score
Experimental group	40	68.30 ± 4.01	94.53 ± 5.33
Control group	40	58.85 ± 3.91	84.48 ± 3.89
*t*		10.671	9.633
*p*		<0.001	<0.001

**Table 4:** Comparison of the incidence of complications in perioperative period (*n*(%)).

Group	*n*	Fracture nonunion	Pressure ulcer	Deep venous thrombosis of lower extremities	Joint stiffness	Total incidence of complications
Experimental group	40	0 (0.00)	1 (2.50)	1 (2.50)	0 (0.00)	5.00 (2/40)
Control group	40	2 (5.00)	3 (7.50)	2 (5.00)	1 (2.50)	20.00 (8/40)
X^2^						4.114
*p*						<0.05

## Data Availability

The data used to support the findings of this study are available on reasonable request from the corresponding author.
